# The Protective Role of Brain CYP2J in Parkinson's Disease Models

**DOI:** 10.1155/2018/2917981

**Published:** 2018-06-26

**Authors:** Yueran Li, Jinhua Wu, Xuming Yu, Shufang Na, Ke Li, Zheqiong Yang, Xianfei Xie, Jing Yang, Jiang Yue

**Affiliations:** ^1^Department of Pharmacology, School of Basic Medical Sciences, Wuhan University, Wuhan 430071, China; ^2^Demonstration Center for Experimental Basic Medicine Education, School of Basic Medical Sciences, Wuhan University, Wuhan 430071, China

## Abstract

CYP2J proteins are present in the neural cells of human and rodent brain regions. The aim of this study was to investigate the role of brain CYP2J in Parkinson's disease. Rats received right unilateral injection with lipopolysaccharide (LPS) or 6-hydroxydopamine (6-OHDA) in the substantia nigra following transfection with or without the CYP2J3 expression vector. Compared with LPS-treated rats, CYP2J3 transfection significantly decreased apomorphine-induced rotation by 57.3% at day 12 and 47.0% at day 21 after LPS treatment; moreover, CYP2J3 transfection attenuated the accumulation of *α*-synuclein. Compared with the 6-OHDA group, the number of rotations by rats transfected with CYP2J3 decreased by 59.6% at day 12 and 43.5% at day 21 after 6-OHDA treatment. The loss of dopaminergic neurons and the inhibition of the antioxidative system induced by LPS or 6-OHDA were attenuated following CYP2J3 transfection. The TLR4-MyD88 signaling pathway was involved in the downregulation of brain CYP2J induced by LPS, and CYP2J transfection upregulated the expression of Nrf2 via the inhibition of miR-340 in U251 cells. The data suggest that increased levels of CYP2J in the brain can delay the pathological progression of PD initiated by inflammation or neurotoxins. The alteration of the metabolism of the endogenous substrates (e.g., AA) could affect the risk of neurodegenerative disease.

## 1. Introduction

Parkinson's disease (PD) is a progressive neurodegenerative disorder characterized by motor symptoms, including bradykinesia with resting tremor, rigidity, and gait disturbance. The major neuropathological findings of PD are the loss of dopaminergic (DA) neurons and the presence of *α*-synuclein-containing aggregates in the substantia nigra (SN). Although the underlying mechanisms remain unknown, putative factors in PD pathogenesis include oxidative stress, proteostasis imbalance, neuroinflammation, environmental toxins, and genetic variants.

Increasing evidence indicates that neuroinflammation is an important contributor to PD pathogenesis and that peripheral inflammation contributes to the initiation and/or progression of the disease by exacerbating and synergizing with neuroinflammation [1]. Astrocytes play vital roles in neuroinflammatory processes in PD [2]. They respond to inflammatory stimulation by producing proinflammatory cytokines both *in vitro* and *in vivo* [3, 4]. Astrocyte-specific overexpression of mutant *α*-synuclein causes widespread astrogliosis, microglial activation, and the degeneration of DA neuron in mice [5]. Reactive astrogliosis has been reported in PD animal models and in the affected brain regions of patients with PD [6]. Astrocytes amplify the inflammatory signals activated by microglia, and uncontrolled neuroinflammation ultimately contributes to neurodegeneration [3, 7]. The injection of lipopolysaccharide (LPS) into the SN induces the progressive, specific, and irreversible loss of DA neurons and the accumulation of *α*-synuclein [8]. The intranigral injection of LPS into the striatum and nigra causes no detectable damage to GABAergic or serotoninergic neurons, suggesting that DA neurons are selectively vulnerable to LPS [9].

In addition to neuroinflammation, oxidative stress is a critical neurotoxic event in the death of DA neurons [10]. Actually, the inflammation and oxidative stress are tightly linked and may be a positive reciprocal feedback loop in the pathophysiological processes of many chronic diseases including PD [11]. Nuclear factor erythroid 2-related factor 2 (Nrf2), a key regulator of the antioxidant system, has been shown to be a therapeutic target for PD. And the genetic association has been previously reported between functional polymorphisms of the Nrf2-encoding *NFE2L2* gene and the risk of Parkinson's disease [12, 13]. The dopamine analog 6-hydroxydopamine (6-OHDA), a typical neurotoxin, produces high levels of reactive oxygen species and causes mitochondrial dysfunction [14]. The injection of 6-OHDA into the striatum causes the progressive loss of nigral DA neurons; however, no *α*-synuclein aggregates were observed in this model [15, 16].

Cytochrome P450 (CYP) is a superfamily responsible for the biotransformation of exogenous and endogenous compounds. The previous study has shown that CYP2J acts as an arachidonic acid (AA) epoxygenase, and epoxidation of AA produces four regioisomeric *cis*-epoxyeicosatrienoic acids (5,6-, 8,9-, 11,12-, and 14,15-EET) [17]. EETs are metabolized into dihydroxyeicosatrienoic acids by soluble epoxide hydrolase [18]. Immunohistochemistry experiments confirm the presence of CYP2J proteins in the neurons of human and rodent brain regions [19]. In the present study, we investigated the protective role of brain CYP2J and possible mechanisms of action in LPS and 6-OHDA PD models.

## 2. Methods

### 2.1. Animals

Male adult Wistar rats weighing 250–300 g, supplied by the Experimental Animal Center (Hubei, China), were kept at room temperature (22°C–25°C) on a 12 h artificial light/dark cycle, with free access to food and water. Animals were allowed to habituate for 7 days prior to use. All procedures were approved by the Animal Care Committee of Wuhan University and complied with the recommendations of the International Association for the Study of Pain [20]. Rat CYP2J3 is the major isoform in the CYP2J subfamily, which shares a high identity of amino acid sequence with human CYP2J2 (>70%) [21].

### 2.2. Plasmid Construction

The fragment encoding *CYP2J2* was cloned into the pcDNA-3.1(+) vector (YouBio Biological Technology Co., Wuhan, China) after the digestion by BamHI/EcoRI (Thermo Scientific, Waltham, MA, USA). The fragment encoding *CYP2J3* was cloned into the pHAGE-CMV-MCS-IZsGreen vector (Stargene SciTech Development Co., Wuhan, China) after the digestion by Xhol/HindIII (Thermo Scientific, Waltham, MA, USA). The fragment encoding primary *miR-340* was cloned into the pcDNA-3.1(−) vector (Invitrogen, Carlsbad, CA, USA) after the digestion by NotI/BamHI (Thermo Scientific, Waltham, MA, USA). All final constructs were verified by DNA sequence analysis.

### 2.3. Lentiviral Vector (LV) Construction

Recombinant lentiviruses were produced by transfecting 293T cells with a viral vector containing the enhanced green fluorescent protein (eGFP) gene, the CYP2J3 expression vector or a control vector, and packing and envelope plasmids (psPAX2 and pMD2.G; Addgene, Cambridge, MA, USA) using Lipofectamine 2000. The virus-containing medium was harvested after 48 and 72 h, then concentrated by a two-step ultracentrifugation procedure after filtration. Titers of the viral vectors used in this study ranged from 1 to 2 × 10^9^ TU/ml.

### 2.4. Surgery and Treatment Procedure

The procedure for implantation of i.c.v. guide cannula was conducted as previously described [22]. The rats were anesthetized by chloral hydrate (300 mg/kg, i.p.) and were secured in a stereotaxic frame (RWD Life Science, Shenzhen, China). The head was shaved, and a 1 mm hole was drilled using a high-speed drill (RWD Life Science, Shenzhen, China). A guide cannula (62003, RWD Life Science, Shenzhen, China) was implanted at 0.5 mm above the right substantia nigra pars compacta (SNpc) (Bregma coordinates: AP, 5.3 mm; ML, 2.0 mm; and DV, 7.8 mm). The insertion cannula for stereotaxic injection protruded 0.5 mm below the tip of the guide cannula. Guide cannula was fixed with acrylic dental cement and three stainless steel screws affixed to the skull. The incision was closed using 5-0 Dysilk. Animals were administered with benzylpenicillin (60 mg/kg, s.c.) after the operation and kept warm until they were awake. Body weights and clinical signs were monitored closely during postsurgical recovery.

Experiment I. A total of 60 rats were randomly divided into the following groups: control group, LPS group, LPS treatment following empty vector transfection, and LPS treatment following LV-CYP2J3 transfection (*n* = 15). LPS (from *Escherichia coli*, serotype O55:B5, Sigma, St. Louis, MO, USA), dissolved in sterile phosphate-buffed saline (PBS), was unilaterally injected (10 *μ*g, 2 *μ*l) into the right SNpc of rats at a rate of 0.2 *μ*l/min by an automatic injector (CMA 402, CMA Microdialysis AB, Sweden) in the CMA 120 System for Freely Moving Animals (CMA Microdialysis AB) [23]. The syringe was left in situ for 5 min. Control animals were injected with sterile PBS. After injection, the syringe was left in situ for 5 min. Rats received unilateral injections of the empty vector or the LV-CYP2J3 vector 3 days before treatment with LPS. One microliter LV was injected for 5 min at a rate of 0.2 *μ*l/min by an automatic injector. Using a fluorescent microscope, the expression of eGFP was used as a visual marker of the injection site and LV transduction.

Experiment II. A total of 40 rats were randomly divided into the following groups: control group, 6-OHDA group, 6-OHDA treatment following empty vector transfection, and 6-OHDA treatment following LV-CYP2J3 transfection (*n* = 10). 6-OHDA (Sigma, St. Louis, MO, USA) was dissolved in sterile saline with 0.2% vitamin C. For the 6-OHDA PD animal model, 6-OHDA (8 *μ*g, 2 *μ*l) was unilaterally injected into the right SNpc of rats. Control animals were injected with the vehicle. Rats received unilateral injections of the control vector or the LV-CYP2J3 vector 3 days before 6-OHDA treatment. One microliter of LV was injected for 5 min at a rate of 0.2 *μ*l/min by an automatic injector. After injection, the syringe was left in situ for 5 min.

### 2.5. Rotational Behavior

The animals were tested for rotational behavior after treatment with the DA agonist apomorphine (0.5 mg/kg, s.c.) dissolved in sterile saline 12 and 21 days after LPS or 6-OHDA injections [24]. Rats were placed in a circular test arena. Rotational activity was measured for 30 min, beginning 5 min after injection, and the number of turns was counted [25].

### 2.6. Immunohistochemistry

Rats were deeply anesthetized and perfused with saline followed by cold 4% paraformaldehyde through the aorta. Brain tissues were quickly removed and postfixed with 4% paraformaldehyde. The samples were embedded in paraffin, and a series of 4 *μ*m sections were cut. Four sections were selected from the SN, and sections from different groups were matched as closely as possible [26]. The sections were incubated with a polyclonal rabbit anti-rat antibody for tyrosine hydroxylase (TH, 1 : 200). After incubation with biotinylated anti-rabbit IgG (1 : 100), the antigen-antibody complex was visualized using the avidin-biotin complex technique (ABC kit, Vector Laboratories, Burlington, Ont., Canada) followed by a reaction with 3,3′-diaminobenzidine and hydrogen peroxide (DAB kit, Vector Laboratories, Burlington, Ont., Canada). TH-positive cells in the lesioned and intact hemispheres were assayed using the ImageJ software to measure a gray scale value within the range of 0–200. Background staining was subtracted, and analysis was performed blinded. The data shown are the percentage of cells relative to the intact SN side.

### 2.7. Immunofluorescence

To investigate the effects of CYP2J on Nrf2 protein levels, brain tissues from both LPS and 6-OHDA PD models were fixed with 4% paraformaldehyde. The SN was embedded in paraffin and cut into 4 *μ*m. After deparaffinization and rehydration of the paraffin sections, antigen retrieval was performed with citrate buffer (0.1 M, pH 6.0) at 95°C for 10 min. The sections were blocked with 3% BSA for 1 h and incubated with a polyclonal rabbit anti-rat CYP2J antibody (1 : 400) and a monoclonal mouse anti-rat Nrf2 antibody (1 : 200). The samples were incubated with the secondary antibodies including a rhodamine-conjugated AffiniPure Goat anti-rabbit IgG for CYP2J (1 : 100) and a Cy3-conjugated AffiniPure Donkey anti-mouse IgG for Nrf2 (1 : 100). Images were analyzed using an Olympus BX51 fluorescent microscope (Olympus Corporation, Tokyo, Japan) equipped with an Olympus Micro DP72 camera. Identical illumination and camera settings were used within each data set.

To investigate the effects of CYP2J on *α*-synuclein accumulation, the SN from the LPS PD model was co-incubated with a monoclonal mouse anti-rat *α*-synuclein antibody (1 : 400) and a polyclonal rabbit anti-rat TH antibody (1 : 200). Then, the samples were incubated with the secondary antibodies which included a rhodamine-conjugated AffiniPure Goat anti-rabbit IgG for TH (1 : 100) and a Cy3-conjugated AffiniPure Donkey anti-mouse IgG for *α*-synuclein (1 : 100).

To investigate the effects of LPS on the p-CREB levels, U251 cells were pretreated with CLI-095 (1 *μ*M) or ST 2825 (20 *μ*M) for 1 h before LPS treatment (1 *μ*g/ml, 24 h). The cells were fixed and permeabilized with 0.5% Triton X-100. Fixed cells were blocked with 3% fetal calf serum for 30 min. The cells were incubated with monoclonal rabbit anti-human p-CREB (S133) antibody and goat anti-mouse alpha tubulin antibody overnight at 4°C. Samples were incubated with fluorescent-labeled goat anti-rabbit IgG and fluorescent-labeled goat anti-mouse IgG in PBS for 1 h at 37°C. Then, the cells were washed twice in PBS and incubated with 4,6-diamidino-2-phenylindole (DAPI) for 5 min.

### 2.8. Cell Culture and Treatment

Human glioma U251 cells were grown in Dulbecco's modified Eagle's medium containing 10% fetal bovine serum. To determine whether CYP2J or AA metabolite plays a role in oxidative stress, U251 cells were transfected with the CYP2J2 expression vector or treated with 14,15-EET (1 *μ*M) and 12-(3-adamantan-1-yl-ureido)dodecanoic acid (AUDA) (1 *μ*M), an inhibitor of soluble epoxide hydrolase. To investigate the mechanism by which LPS regulates CYP2J, U251 cells were pretreated with a specific TLR4 inhibitor (CLI-095, 1 *μ*M) or a specific MyD88 inhibitor (ST 2825, 20 *μ*M) for 1 h before LPS treatment (1 *μ*g/ml, 24 h).

### 2.9. Real-Time RT-PCR

Total RNA was isolated using the TRIzol reagent (Invitrogen, Carlsbad, CA, USA). cDNA was synthesized using a cDNA Synthesis Kit (Toyobo, Osaka, Japan) for first-strand synthesis. All real-time PCR reactions with SYBR Green (Toyobo, Osaka, Japan) were performed on a CFX connect real-time PCR detection system (Bio-Rad, Hercules, CA, USA). For miR-340 detection, a small RNA-specific stem-loop RT primer was used as follows: 5-GTCGTATCCAGTGCGTGTCGTGGAGTCGGCAATTGCACTGGATACGACAATCAG-3′. The primers for PCR are listed in Additional file 1 (Table S1). Human GAPDH was used for the normalization of relative expression levels, and U6 was used to normalize the relative expression of miR-340. Gene expression levels were calculated using the 2^−ΔΔCT^ method relative to internal controls.

### 2.10. Immunoblotting

The pellets of cells were lysed using RIPA lysis buffer. For the detection of Nrf2 proteins, 20 *μ*g of total proteins from U251 cells were separated by SDS-polyacrylamide gel electrophoresis (4% stacking and 10% resolving gels) and then transferred onto PVDF membranes. These membranes were incubated for 2 h with a polyclonal rabbit anti-human Nrf2 antibody (1 : 1000). The protein levels of Nrf2 were normalized to *β*-actin (1 : 1000) to control the loading efficiency. The immunoblots were visualized using chemiluminescence followed by exposure to autoradiography films and analyzed using Gel Documentation & Analysis Systems (Beijing Liuyi Instrument, Beijing, China). The relative density of each band was expressed in arbitrary density units after subtracting the background.

### 2.11. Chromatin Immunoprecipitation (ChIP) Assay

The ChIP kit (EpiGentek Group Inc., Brooklyn, NY, USA) was used to determine the binding profile of *CYP2J2* genes with p-CREB protein in cells pretreated with or without CLI-095 (1 *μ*M) or ST 2825 (20 *μ*M) for 1 h before LPS treatment (1 *μ*g/ml, 24 h). Briefly, the cross-linked chromatin from the nuclear fraction was sheared into fragments of the proper length by sonication according to the manufacturer's protocol. The chromatin concentration was measured, and approximately 10% of the chromatin was retained as input material. The chromatin solution was immunoprecipitated with rabbit anti-human p-CREB (S133) antibody (1 : 100) or non-immune mouse IgG as a negative control. The number of cycles used for PCR amplification were within the linear range (primers are listed in Table S1), and PCR products were resolved on a 2% agarose gel. The band intensities were quantified using an AutoChemi Imaging System (UVP LLC, Upland, CA, USA).

### 2.12. Materials

LPS (cat. number L2880) and 6-OHDA (cat. number H116) were purchased from Sigma (St. Louis, MO USA), 14,15-EET were purchased from Cayman Chemical Co. (cat. number 50651, Ann Arbor, MI), apomorphine (cat. number HY-12723A) and ST 2825 (cat. number HY-50937) were purchased from MedChem Express (Princeton, NJ, USA), and CLI-095 was purchased from InvivoGen (cat. number tlrl-cli95, San Diego, CA, USA).

Primary antibodies to TH (cat. number ab112), Nrf2 (cat. number ab89443), *α*-synuclein (cat. number ab1903), and p-CREB (S133) (cat. number ab32096) were purchased from Abcam (Cambridge, MA, USA). Primary antibodies to CYP2J were purchased from Merck Millipore (cat. number ABS1605, CA, USA). Primary antibodies to TH were purchased from GeneTex Inc. Irvine (cat. number GTX113016, CA, USA). Primary antibodies to alpha-tubulin were purchased from Proteintech (cat. number 66031-1-lg, Chicago, IL, USA). Primary antibodies to *β*-actin were purchased from Santa (cat. number sc-8432, Santa Cruz, CA, USA). Rhodamine-conjugated AffiniPure Goat anti-rabbit IgG was purchased from Kerui Biotechnology Co. (cat. number 100428, Wuhan, China) and DyLight 405 Donkey anti-mouse IgG was purchased from Antgene (cat. number ANT080, Wuhan, China). FITC-conjugated AffiniPure Goat anti-rabbit IgG (cat. number AS1110) and CY3-conjugated AffiniPure Goat anti-mouse IgG (cat. number AS1111) were purchased from Aspen Biological (Wuhan, China).

Dulbecco's modified Eagle's medium (DMEM) was purchased from HyClone (Rockford, IL, USA); reduced serum medium Opti-MEM was purchased from Gibco (Carlsbad, CA, USA). Lipofectamine 2000 was purchased from Invitrogen (Carlsbad, CA, USA). Fetal bovine serum (FBS) was purchased from Zhejiang Tianhang Biotechnology Co. (Zhejiang, China). Other materials were purchased from standard suppliers or as indicated in the text.

### 2.13. Statistical Analysis

All data are expressed as arithmetic mean with a standard error of the mean (SEM). The normalized mRNA levels of genes from cells and rat brain tissue were expressed as arbitrary density units. Results from the ChIP assay were expressed as arbitrary density units and normalized to input levels. Data were obtained from at least five separate experiments. One-way ANOVA was used to test for differences among the groups and was followed by the least significant difference post hoc test. A value of *p* < 0.05 was considered significant.

## 3. Results

### 3.1. LPS Downregulated CYP2J Levels via the TLR4-MyD88 Signaling Pathway in U251 Cells

Our previous study showed that brain CYP2J2 is the target gene of CREB in astrocytes [17]. Compared with controls, mRNA levels of CYP2J2 and CREB were decreased by 67.4% and 34.8%, respectively, after LPS treatment for 24 h (Figure 1(a)). The LPS-induced inhibition of CYP2J2 and CREB mRNA levels was abolished by CLI-095 (a specific TLR4 inhibitor) and partly attenuated by ST 2825 (a specific MyD88 inhibitor) compared with the LPS group. Immunofluorescence data showed that CLI-095 and ST 2825 attenuated LPS-induced decreases in the p-CREB protein level in cells (Figure 1(b)). ChIP data showed that p-CREB proteins bound to the *CYP2J2* promoter at −1426 to −1405 bp. Compared with the control, binding of the p-CREB protein to the *CYP2J2* promoter was decreased by 50% following LPS treatment; however, decreased binding of the p-CREB protein to the *CYP2J2* promoter induced by LPS was attenuated by CLI-095 and ST 2825 (Figure 1(c)). These data suggest that the TLR4-MyD88 signaling pathway is involved in the regulation of CYP2J via CREB following treatment with LPS.

### 3.2. CYP2J-Dependent Metabolites Upregulated Antioxidative Genes via miR-340

Compared with controls, CYP2J2 overexpression significantly increased both the mRNA and protein levels of Nrf2 in U251 cells (Figures 2(a)–2(c)). The mRNA levels of genes related to mitochondrial oxidative defense (SOD1, CAT, and GPX1) in astrocytes were significantly elevated by CYP2J2 overexpression compared with controls; however, no changes were observed in the mRNA levels of genes related to endoplasmic reticulum stress, including MANF, PERK, IRE1*α*, and ATF6 (data not shown). Compared with controls, the level of miR-340 mRNA was significantly decreased following CYP2J2 overexpression (Figure 2(d)). Western blotting and real-time RT-PCR revealed that miR-340 targeted Nrf2 expression in astrocytes (Figures 2(e)–2(g)). Following 14,15-EET and/or AUDA (a soluble epoxide hydrolase inhibitor) treatment of U251 cells, miR-340 and Keap1 were downregulated; however, genes related to mitochondrial oxidative defense were upregulated including Nrf2, SOD1, CAT, and GPX1 (Figures 2(h)–2(m)).

### 3.3. CYP2J Transfection Protected Dopaminergic Neurons in the LPS PD Animal Model

The accumulation of *α*-synuclein was observed after LPS treatment for 12 and 21 days (Figure 3(a)); however, CYP2J transfection attenuated the LPS-induced accumulation of *α*-synuclein. Compared with the control, the number of DA neurons was decreased by 75.5% after stereotaxic injections of LPS for 21 days (Figures 3(b) and 3(c)); however, DA neurons remaining in the SNpc of rats transfected with the CYP2J expression vector were increased by 2.1-fold compared with the LPS group. Compared with LPS-treated rats, the number of rotations in rats transfected with the CYP2J expression vector was decreased by 57.3% at day 12 and 47.0% at day 21 after LPS treatment (Figures 3(d) and 3(e)).

### 3.4. CYP2J Transfection Upregulated Genes Related to Mitochondrial Oxidative Defense in the LPS PD Animal Model

The effect of CYP2J expression on Nrf2 protein levels was investigated by fluorescent immunocytochemistry. Levels of Nrf2 protein were elevated in cells with high levels of CYP2J3 after LPS treatment for 12 and 21 days compared with the LPS group (Figures 4(a) and 4(b)). Compared with the control, mRNA levels of CREB and CYP2J3 in the SN were decreased by 31.0% and 45.6%, respectively, following LPS treatment for 21 days, but miR-340 mRNA levels were increased by 2.5-fold, and levels of genes related to mitochondrial oxidative defense were decreased. Compared with the LPS group, the mRNA levels of Nrf2, SOD1, CAT, and GPX1 in rat SN transfected with the CYP2J3 expression vector were increased by 6.0-, 2.6-, 3.2-, and 3.2-fold, respectively, and miR-340 mRNA levels were decreased by 47.7% (Figures 4(c) and 4(d)).

### 3.5. CYP2J Transfection Protected Dopaminergic Neurons in the 6-OHDA PD Animal Model

Compared with the control, the number of DA neurons decreased by 74.8% after treatment with 6-OHDA for 21 days; however, in the SNpc of rats transfected with the CYP2J expression vector, the number of DA neurons increased by 2.4-fold compared with the 6-OHDA and pHAGE groups (Figures 5(a) and 5(b)). Compared with 6-OHDA-treated rats, rotations in rats transfected with the CYP2J3 expression vector were decreased by 59.6% at day 12 and 43.5% at day 21 after 6-OHDA treatment (Figures 5(c) and 5(d)).

### 3.6. CYP2J Transfection Upregulated Genes Related to Mitochondrial Oxidative Defense in the 6-OHDA PD Animal Model

Compared with the 6-OHDA group, Nrf2 protein levels were elevated in cells with high levels of CYP2J3 after 6-OHDA treatment for 12 and 21 days indicated by fluorescent immunocytochemistry (Figures 6(a) and 6(b)). Compared with the control, CREB and CYP2J3 mRNA levels in the SN decreased by 16.5% and 55.2%, respectively, following 6-OHDA treatment (Figure 6(c)). However, the 6-OHDA-induced inhibition of genes related to mitochondrial oxidative defense was attenuated by transfection with CYP2J3. Compared with the control, mRNA levels of Nrf2, SOD1, CAT, and GPX1 in rat SN transfected with the CYP2J3 expression vector were increased by 8.7-, 4.9-, 12.9-, and 6.5-fold, respectively, and miR-340 mRNA levels were decreased by 48.8% (Figure 6(d)).

## 4. Discussion

This is the first demonstration that brain CYP2J plays a protective role in PD models induced by inflammation or oxidative stress. We showed that (i) CYP2J3 transfection significantly attenuated LPS- or 6-OHDA-induced behavioral impairment and the loss of DA neurons in the SN; (ii) the TLR4-MyD88 signaling pathway was involved in the downregulation of brain CYP2J induced by LPS; and (iii) both CYP2J transfection and 14,15-EET activated the Nrf2-antioxidant response element (ARE) pathway via the inhibition of miR-340. These data indicate that AA metabolites catalyzed by brain CYPs may affect the mitochondrial oxidative defense system.

A growing body of basic research shows that the Nrf2-ARE pathway plays a protective role in both toxin-induced and transgenic mouse models of PD [27]. Following oxidative stress, Nrf2 is released from Keap1, translocates into the nucleus, and binds with the ARE of antioxidant genes. Our data showed the activation of the Nrf2-ARE pathway by 14,15-EET treatment in astrocytes, which is consistent with a previous report that 14,15-EET treatment significantly increased the accumulation of Nrf2 in lung epithelial cells [28]. The downstream target genes of Nrf2 related to mitochondrial oxidative defense were upregulated following CYP2J transfection, suggesting that Nrf2 can prevent the damage to mitochondria from oxidant injury. The previous study showed that the isolated mitochondria from the myocardium of Nrf2 deficiency mice were more sensitive to mitochondrial membrane permeability transition and swelling compared with the samples from the wild-type mice (Nrf2 protects mitochondrial decay by oxidative stress). The induction of Nrf2 attenuated microglia-induced inflammation in the hippocampus of LPS-treated mice as determined by reduced inducible NO synthase (iNOS) levels and attenuated the production of proinflammatory cytokines IL-6 and TNF-*α* [29]. Nrf2 overexpression inhibited RAC1-dependent activation of nuclear factor-*κ*B (NF-*κ*B), indicating a cross-talk between Nrf2 and NF-*κ*B pathways [30]. The activation of the Nrf2-ARE pathway following CYP2J overexpression or the treatment of EETs may also inhibit the NF-*κ*B signaling pathway. Recently, Nrf2 was identified as a regulator of the expression of autophagy genes [31, 32]. Our data showed the downregulation of Nrf2 and its downstream genes in both the LPS and 6-OHDA PD models, suggesting that the Nrf2-ARE pathway is associated with both neuroinflammation and oxidative stress. Nrf2 may be a suitable pharmacological target for the treatment of PD [27].

Cardiovascular EETs have been reported to inhibit reactive oxygen species, the inflammatory reaction, vascular smooth muscle migration, and enhancement of the fibrinolytic pathway [33]. Our data suggest that EETs may play a protective role in PD. A previous study showed that sEH deficiency or inhibition attenuated MPTP-induced dopamine neuron loss and behavioral deficits [34]. Our data showed that 14,15-EET decreased miR-340 levels and that the LPS-induced elevation of miR-340 levels was attenuated by CYP2J overexpression. The overexpression of miR-340 decreased Nrf2 mRNA levels in neural cells, which is consistent with a previous study showing that miR-340 directly targets Nrf2 mRNA in hepatocytes [35].

The TLR4-MyD88 signaling pathway is involved in decreasing CYP2J in astrocytes via CREB following LPS treatment. Previous studies have shown that *α*-synuclein secreted from neurons induced a TLR4-dependent inflammatory response in primary astrocyte cultures [36]. The accumulation of *α*-synuclein in astrocytes following the overexpression of mutant *SNCA* (encoding *α*-synuclein) under an astrocyte-specific promoter resulted in the degeneration of DA neurons in the SNpc and the ventral tegmental area (VTA), as well as the onset of a movement disorder [37]. Data from this study indicate that activation of the TLR4 signaling pathway results in the downregulation of antioxidative systems in astrocytes via inhibition of brain CYP2J. Alterations of the CYP2J-dependent metabolism of endogenous substrates may attenuate the LPS- or 6-OHDA-induced loss of DA neurons and accumulation of *α*-synuclein in the SN.

In conclusion, our data demonstrated that the elevated CYP2J levels strengthen the antioxidative defense system by altering miRNA profiles within the brain. This suggests that the alteration of the metabolism of the endogenous substrates (e.g., AA) could affect the risk of neurodegenerative disease induced by neuroinflammation or neurotoxins. The CYP2J-mediated metabolites may activate the Nrf2-ARE pathway and delay PD progression by ameliorating mitochondrial dysfunction.

## Figures and Tables

**Figure 1:** The TLR4-MyD88 signaling pathway was involved in the inhibition of CYP2J2 levels by LPS treatment in U251 cells. Compared with the control, LPS treatment decreased CYP2J and CREB mRNA levels in cells (a). The LPS-induced inhibition of CYP2J2 and CREB mRNA levels was abolished by CLI-095 and attenuated by ST 2825. Moreover, CLI-095 and ST 2825 attenuated the LPS-induced decrease in p-CREB protein levels in cells (b). ChIP data shows that the LPS-induced decrease of p-CREB protein binding to the *CYP2J2* promoter by LPS was attenuated by CLI-095 and ST 2825 (c). Data were analyzed by one-way ANOVA. The data are mean ± SEM; *n* = 5, ^∗^ *p* < 0.05, ^∗∗^ *p* < 0.01, and ^∗∗∗^ *p* < 0.001 compared with respective controls.

**Figure 2:** Astrocytic CYP2J upregulated the antioxidative system via the inhibition of miR-340 in U251 cells. Compared with controls, mRNA levels of Nrf2, SOD1, CAT, and GPX1 were increased in cells following transfection with the CYP2J2 expression vector (a); moreover, Nrf2 protein levels were increased indicated by Western blotting (b and c). The level of miR-340 mRNA was decreased following transfection with CYP2J2 (d) compared with the control. Nrf2 mRNA (e) and protein (f and g) levels were decreased following miR-340 transfection. Compared with the controls, 14,15-EET and/or AUDA (a soluble epoxide hydrolase inhibitor) treatment decreased the mRNA levels of miR-340 (h) and Keap1 (j) but increased mRNA levels of Nrf2 (i), SOD1 (k), CAT (l), and GPX1 (m) in U251 cells. Data were analyzed by one-way ANOVA. The data are mean ± SEM; *n* = 5, ^∗^ *p* < 0.05, ^∗∗^ *p* < 0.01, and ^∗∗∗^ *p* < 0.001 compared with respective controls.

**Figure 3:** The effects of CYP2J transfection on the loss of dopaminergic (DA) neurons in the SN and behavioral impairment in the LPS PD animal model. Fluorescent immunocytochemistry data shows the accumulation of *α*-synuclein (blue) in tyrosine hydroxylase positive neurons (red) after LPS treatment for 12 and 21 days (a); however, CYP2J transfection attenuated the LPS-induced accumulation of *α*-synuclein. Immunohistochemistry staining shows the loss of DA neurons in the SN after LPS treatment (b). There were an increased number of DA neurons remaining in the SNpc of rats transfected with the CYP2J3 expression vector compared with the LPS group (c). Compared with LPS-treated rats, the number of rotations by rats with high CYP2J3 levels was decreased on day 12 (d) and day 21 (e) after LPS treatment. Data were analyzed by one-way ANOVA. The data are mean ± SEM; *n* = 15, ^∗^ *p* < 0.05 compared with respective controls.

**Figure 4:** Changes in genes related to mitochondrial oxidative defenses in the LPS PD animal model. Fluorescent immunocytochemistry data shows reduced levels of Nrf2 (blue) and CYP2J3 (red) protein in rats treated with LPS for 12 and 21 days (a). Nrf2 protein levels were increased following transfection with the CYP2J3 expression vector (b). Compared with the control, mRNA levels of CREB and CYP2J3 were decreased following LPS treatment (c) but miR-340 mRNA levels were increased (d). Compared with the LPS group, the LPS-induced inhibition of Nrf2, SOD1, CAT, and GPX1 mRNA levels was attenuated by transfection with CYP2J3 (d). Data were analyzed by one-way ANOVA. The data are mean ± SEM; *n* = 5, ^∗^ *p* < 0.05, ^∗∗^ *p* < 0.01, and ^∗∗∗^ *p* < 0.001 compared with respective controls.

**Figure 5:** The effects of CYP2J3 transfection on the loss of dopaminergic (DA) neurons in the SN and behavioral impairment in the 6-OHDA PD animal model. Immunohistochemistry staining showed the loss of DA neurons in the SN after 6-OHDA treatment (a). The dopaminergic neurons left in SNpc from the rats transfected with CYP2J3 expression vector were increased, compared with the 6-OHDA group (b). Compared with 6-OHDA-treated rats, the number of rotations in rats with high CYP2J3 levels was decreased at day 12 (c) and day 21 (d) after 6-OHDA treatment. ^∗∗∗^ *p* < 0.001 compared with respective controls.

**Figure 6:** Changes in genes related to mitochondrial oxidative defenses in the 6-OHDA PD animal model. Fluorescent immunocytochemistry data shows reduced levels of Nrf2 (blue) and CYP2J3 (red) protein in rats treated with 6-OHDA for 12 and 21 days (a). Nrf2 protein levels were increased following transfection with the CYP2J3 expression vector (b). Compared with the control, mRNA levels of CREB and CYP2J3 were decreased by 6-OHDA treatment (c). The inhibition of Nrf2, SOD1, CAT, and GPX1 mRNA levels following 6-OHDA treatment was attenuated by transfection with CYP2J3, compared with the 6-OHDA group (d). Data were analyzed by one-way ANOVA. The data are mean ± SEM; *n* = 5, ^∗^ *p* < 0.05, ^∗∗^ *p* < 0.01, and ^∗∗∗^ *p* < 0.001 compared with respective controls.

## Data Availability

The data used to support the findings of this study are available from the corresponding author upon request.

## Abbreviations

AA: Arachidonic acid
ANOVA: Analysis of variance
AUDA: 12-(3-Adamantan-1-yl-ureido)dodecanoic acid
CYP2J2: Cytochrome P450 2J2
DA: Dopaminergic
EETs: *cis*-Epoxyeicosatrienoic acids
LPS: Lipopolysaccharide
LV: Lentiviral vector
miRNA: MicroRNA
6-OHDA: 6-Hydroxydopamine
PBS: Phosphate-buffed saline
PD: Parkinson's disease
SN: Substantia nigra
SNpc: Substantia nigra pars compacta
TH: Tyrosine hydroxylase
TLR4: Toll-like receptor 4
3'-UTR: 3′-Untranslated region
VTA: Ventral tegmental area.

## Additional Points

*Declaration of Transparency and Scientific Rigour*. This declaration acknowledges that this paper adheres to the principles for transparent reporting and scientific rigour of preclinical research recommended by funding agencies, publishers, and other organizations engaged with supporting research.

## Supplementary Materials

Supplementary Materials Primers used in this study are listed in Table S1.
